# Discrete Dynamic Modeling of Learner Behavior Analysis in Physical Education Teaching

**DOI:** 10.1155/2022/4620599

**Published:** 2022-04-12

**Authors:** Jia Shi, Jun Sun, Zhonghua Zheng

**Affiliations:** Department of Sports, Central China Normal University, Wuhan, Hubei 430070, China

## Abstract

With the advent of the big data era, the combination of information technology and education has become an important way for the development of the industry. The large-scale realization of teaching tasks under the background of information data requires the prediction and analysis of learners' characteristics, behavior, and development trend. Based on the above situation, this paper uses discrete dynamic modeling technology in big data environment to study the learners' behavior in physical education teaching. By quantifying the learning process data, the feature points of each learner are extracted to realize the personalized construction of dynamic learning data. Due to the rapid development of network technology, we mainly analyze the online education platform and explore the influencing factors of learners' behavior characteristics from many aspects. Finally, it carries out dynamic modeling and prediction for physical education learners from the aspect of achievement change, uses the grey model to build the achievement change system, and combines the dynamic modeling technology to reflect the development trend of achievement. The results show that the main factor affecting learners' behavior change in physical education is video learning. Most students are passive and lack initiative in the learning process. Discrete dynamic modeling technology can improve the accuracy of predicting student achievement changes and provide effective data for the research content.

## 1. Introduction

With the continuous development of the information age, the big data model has become a common data source in many fields (Lin et al., 2021) [1]. Information and data play an important role in human life. In the development of education, the traditional classroom teaching mode has gradually shifted to the modern teaching mode (Zhu et al., 2021) [2]. Using data information to solve the problems encountered in the educational process has become the norm (Cai and Lin, 2021) [3]. In the research of learner behavior analysis and learner feature extraction, the error impact caused by massive data is very obvious. We need to use a series of means to simplify data and extract hidden useful information from large-scale information (Yan et al., 2021) [4]. The ultimate goal is to help teachers accurately analyze students' learning and form targeted teaching methods. At the same time, it can also help learners improve their learning ability and change the traditional single learning method (Shi and Hao, 2021) [5]. For the analysis of learners in the field of sports, it mainly explores from the aspects of intelligence, personalization, and online education. Due to the particularity of sports, the teaching environment needs suitable places as support. Therefore, many problems have been encountered in the transformation of education model (Liao et al., 2021) [6].

For the transformation of physical education teaching mode, we have added many products under big data technology to our teaching methods, using virtual reality technology as an implementation way of online integrated teaching (Zhang and Ge, 2021) [7]. Using virtual reality products in network teaching allows students to experience the immersive teaching environment. This way can improve students' interactive ability and information exchange ability in sports activities (Wang 2020) [8], realizing three-dimensional physical education through touch, hearing, vision, and other senses. Finally, the online learning students are analyzed for learner behavior, mainly using discrete dynamic modeling technology in the context of big data (Zeng et al., 2020) [9]. This technology is used to solve the errors and storage difficulties caused by dynamic growth in the construction of data integration. Learner behavior analysis is the key content of educational research. The traditional research methods mainly use neural network algorithm and deep learning algorithm. Most of this research technology is in the static data environment and is studied from a certain perspective (He and Li, 2020) [10]. In fact, the changes of students' characteristics and behavior are in a dynamic mode, and the data changes are uncertain and dynamic as a whole. Therefore, in the analysis of learners' behavior, we mainly use discrete dynamic modeling technology to explore. We control students' learning styles and rules and study the factors affecting learners' behavior changes from many aspects. Finally, the overall performance of learners is dynamically predicted to obtain the optimal education model.

This paper analyzes the changing trend of learners' behavior in physical education teaching and its influencing factors on performance. This paper mainly discusses the application of data mining in learner behavior analysis and dynamic data processing. Innovative contributions include extracting students' key feature points by quantifying learning process data and providing learners with personalized learning strategies. Compared with the traditional learner behavior analysis model, discrete dynamic modeling can deal with the dynamic information in different environments and improve the overall accuracy of the model. Using the dynamic modeling method, this paper constructs the development and change model of sports performance and tests the results of the model. The error coefficient and accuracy of students' performance change are analyzed in the model. The results show that the discrete dynamic modeling of learner behavior analysis can help teachers effectively obtain students' learning state and learning effect.

This paper is mainly divided into three parts. The first part briefly describes the research status of learner behavior analysis and feature analysis, as well as the application background of discrete dynamic modeling technology. In the second part, firstly, the data mining algorithm is used to obtain student behavior data, and the differences between traditional modeling technology and discrete dynamic modeling technology are compared. Discrete dynamic modeling technology is used to analyze the behavior changes of physical education learners and build an intelligent learning guidance system. Finally, the grey model of learners' performance data in physical education teaching is constructed, and the discrete dynamic modeling is used to predict the change trend of performance. The third part first analyzes the results of the research on the behavior analysis and modeling of sports learners and analyzes the factors affecting the change of learners' behavior. Finally, the results of the prediction model of physical education learners' performance are analyzed.

## 2. Related Work

The research on learner behavior analysis is mainly applied to classroom teaching. Firstly, collect the behavior data generated by students in the learning process, compare the teaching methods, and analyze the interaction between the two (Bi and Zhao, 2015) [11]. The obtained data will be processed and finally fed back to the classroom. Teachers improve teaching methods and optimize students' learning atmosphere by analyzing the results. In order to effectively predict the learning effect, many educational researchers extract the key feature point data according to the learning behavior pattern and construct the prediction model combined with the Bayesian algorithm in discrete dynamic modeling. The experiment mainly verifies the notion that learner behavior analysis can have good prediction effect. In Bayesian algorithm, the weight coefficient and correlation analysis are used to construct the prediction model, identify learners' status, and analyze the main factors affecting performance changes. The main purpose of studying the changes of learners' behavior in teaching in colleges and universities is to analyze students' learning status and carry out personalized teaching setting and intelligent guidance (Mu, 2021) [12].

Most colleges and universities in the United States collect the information data generated in the learning process, mainly to obtain teachers' teaching data and students' feedback data (Wang et al., 2021) [13]. The above information is used to help teachers optimize their teaching methods. By analyzing students' performance score, learning progress, learning effect, and learning style characteristics, this paper predicts whether the learners' whole learning environment is in a normal state. This kind of learner behavior analysis can help teachers quickly solve the problem of students' slack and obtain negative students' personal data. Through information processing, the corresponding intelligent learning methods are matched, combined with targeted optimization of teaching, to improve students' learning experience.

British universities began to monitor and study students' learning process at the end of the nineteenth century. At that time, the technical conditions were poor, and the analysis did not achieve good results (Deepak et al., 2019) [14]. With the rapid development of the information age, British education researchers use data mining and dynamic modeling technology to obtain and process students' learning data. It also makes an effective prediction for the trend of academic achievement. Finally, the analyzed data are fed back to the teaching process, which changes the traditional education model.

The research on online learning behavior patterns in Germany mainly predicts students' performance through identification, classification, diagnosis, and analysis (AbdEllatif et al., 2018) [15]. In the learner behavior model, the education system is constructed by extracting the student behavior sequence, which provides help for the design of the teaching system, using mobile data such as learning duration to analyze students' learning status, compare key behavior sequences, and accurately analyze the factors affecting students' performance. Based on the current situation of learner behavior analysis in the above countries, this paper mainly analyzes the physical education model. This paper studies the factors affecting the change of students' performance in physical education teaching, uses discrete dynamic modeling to construct learners' behavior analysis system, and explores the state change of students in physical education teaching.

## 3. Methodology

### 3.1. Research on Discrete Dynamic Modeling of Learner Behavior Analysis in Physical Education Platform

With the development of computer science, pulse technology, microprocessor, and digital element components, a large number of systems in biology, ecology, aviation, aerospace, economy, and engineering control need to be described by discrete-time systems. When the continuous time system is analyzed and simulated by computer, it also needs to be discretized and then processed. With the expansion of the research field of system theory and the wide popularization and application of computer technology, discrete control system theory has developed rapidly and become an important part of control theory. Discrete system theory plays an important role in the fields of automatic control engineering, communication, radar technology, biology, power system, and nuclear physics. There are essential differences in the description of discrete systems and continuous systems, but there are similarities in analysis and research. Many concepts and research methods in continuous time systems can also be extended and applied to discrete systems.

With the exploration of students' learning analysis technology, more and more educational researchers begin to pay attention to the changes of learners' behavior. Many researchers have proposed a new way to explore learning behavior, that is, to transform and mine the behavior between learning associations. The sequence of behavior characteristics constructs a stable behavior analysis system. The learner behavior analysis system can reflect the time sequence of students' learning behavior, reflect the characteristics between individual and whole learners from a wide-angle perspective, and help teachers to effectively diagnose and improve the differences between different students. In physical education, we need to pay attention to the changes of learners' dynamic operation sequence and mine and extract students' feature points. Finally, the feature point information is identified for online learning pattern simulation, and the system model is constructed according to the original dynamic behavior sequence. The behavior analysis of physical education learning can provide data support for students' learning environment and final performance prediction. This paper constructs a system framework for the online learning behavior model, mainly including the behavior sequence of goals in sports, students' key action events, and behavior changes. Descriptive means are used to identify students' behavior characteristics and complete the preliminary construction of the system model. The framework of learner behavior analysis model is shown in Figure 1.

As can be seen from Figure 1, the behavior mode is mainly composed of description analysis, diagnosis result analysis, and prediction analysis. Through the exploration of all aspects of students, a circular model is formed, extracting the characteristics of target activities from the process of target activities is the basis for analyzing target activities. Firstly, the logical regression algorithm is used to analyze and process the behavior data generated by learners, and the function variables and data loss variables are constructed:

(1) $$\begin{array}{c} P\left(y=1|x\right)=\sigma \left(wx+b\right)=\frac{e^{wx+b}}{e^{wx+b}+1},\\ P\left(y=1|x\right)=1-\sigma \left(wx+b\right)=\frac{1}{e^{wx+b}+1}. \end{array}$$

The above formula can obtain the function value after data processing and the data value lost in the analysis process. When exploring the correlation between learning behavior and result analysis, we use the correlation coefficient of linear regression. The calculation method is as follows:

(2) $$\begin{array}{c} r=\frac{\sum_{i=1}^{n}\left(X_{i}-\bar{X}\right)\left(Y_{i}-\bar{Y}\right)}{\sqrt{{\sum_{i=1}^{n}\left(X_{i}-\bar{X}\right)}^{2}\sqrt{\sum_{i=1}^{n}{\left(Y_{i}-\bar{Y}\right)}^{2}}}}. \end{array}$$

Among them, the value range of correlation coefficient *r* is between positive and negative 1. When the function value is positive, the two variables have correlation. In physical education, the way to study the change of behavior sequence should be analyzed from the perspective of students' movement change. Through the state of students' learning process and the behavior data generated by the online platform, the frequency of students' behavior and activity in different age groups were calculated. Secondly, all learners are classified and analyzed according to the change of feature sequence. Classification and characterization can be used to show the particularity between different groups. Dynamic changes often occur in the processing of students' personal data, for example, replacing and deleting personal data. This situation will also lead to the repetition of historical traces and affect the accuracy of prediction results. Therefore, this paper proposes discrete dynamic modeling technology as a method to build system model. Learner behavior analysis modeling is the process of realizing personalized teaching. The performance of each student in different environments also determines the trend of the overall data. The key feature points of learners are extracted by quantifying student data, and finally the construction of dynamic modeling is realized. Since this process is a random discrete dynamic state, in order to summarize most of the key characteristics and time series changes, this paper adopts a three-stage dynamic modeling path, and the specific process is shown in Figure 2.

As can be seen from Figure 2, the research expresses the behavior analysis and modeling path of physical education learners, which is completed in three stages: quantification of learning data, feature analysis and extraction, and finally recommendation of personality learning methods. Each student will be affected by many factors in different environments, such as learning ability, cognitive level, learning efficiency, and adaptability. In order to analyze the time dimension of learners' behavior change, we use Bayesian network for evolutionary analysis in various places of physical education teaching. The learning process of middle school students in physical education teaching environment is dynamically modeled and evolved, and the personality feature points are extracted. It has made an effective contribution to improving the learning efficiency of middle school students.

Finally, the student feature points after discrete dynamic modeling and analysis are uniformly classified, the repeated links in the data are simplified, and an intelligent guidance system for physical education teaching is formed. Through the analysis of physical education learners' behavior, intelligent guidance can provide targeted learning strategies for each student, promoting students to obtain suitable learning resources in specific ways. With the support of the online platform, learning resources have also been expanded to images, videos, virtual reality scenes, and so on. Because there are spatial attributes such as sparsity and structure between student behaviors, it is necessary to simplify the combination of feature points of data variables. Therefore, discrete dynamic modeling can realize the data processing function under multiangle correlation. For students with different learning environments and learning methods, we comprehensively explore their learning time, learning speed, and learning methods. Combined with discrete dynamic modeling analysis, a behavior inquiry model of physical education learners is formed. It can realize personalized learning strategy recommendation for students from various aspects and automatically make dynamic adjustment according to learners' feedback information.

### 3.2. Research on Student Achievement Prediction Modeling under the Analysis of Learners' Behavior Data in Physical Education Teaching

In physical education teaching activities, the time series prediction method is basically used to predict the change of individual sports performance. According to the time-varying growth coefficient of activity scores as data, mathematical modeling is selected for trend analysis. This situation can easily lead to the expansion of the factors affecting students' sports performance, and the result data is easy to be unknown and fuzzy. Therefore, in the change of learners' behavior in physical education teaching, the prediction of achievement first selects the mathematical model for analysis. This paper focuses on grey model prediction, combined with discrete dynamic modeling technology, to explore the changes of physical education learners' behavior and achievement.

The content of grey model theory is that whether the data is complex or not, it is interrelated, orderly, and in the overall scope. The characteristics of the data cannot use the original sequence model, because the original prediction method cannot accurately calculate the processed data information for the irregular sports results. Firstly, the mined data is used to process the score series in order to provide basic data for subsequent discrete modeling. The set variables are defined as follows:

(3) $$\begin{array}{c} Y_{0};Y_{0}\left(1\right),\ldots ,Y_{0}\left(i\right),\ldots . \end{array}$$

The above formula is used to represent the time-varying performance series. The new sequence formed by accumulating the data is

(4) Y11=∑i=1iYi0

where *Y*_0_(*i*) is the definition of continuous change in the data sequence formed by accumulation. According to the calculation results, we find that the data show discrete changes, and the generated weighted values rise monotonically. The overall randomness of the data has decreased, which is convenient for us to optimize the accuracy of student performance prediction. General models are measured in stages. For the change of sports performance, we set the corresponding generated value about single data. Further considering the discrete change of numerical value, the performance trend is basically in a stable state. This model is a differential calculation equation:

(5) $$\begin{array}{c} \frac{\text{d}Y_{1}\left(t\right)}{\text{d}t}-KY_{1}\left(t\right)=\beta . \end{array}$$

The above formula is equivalent to

(6) $$\begin{array}{c} \frac{\text{d}Y_{1}\text{d}/\text{d}t}{Y_{1}\text{d}}=K+\frac{\beta }{Y_{1}\text{d}}. \end{array}$$

Among them, *K* and *β* are the determined values in the achievement sequence vector in sports, and *K* is the growth efficiency in the cumulative data. We can customize the initial conditions and get the solution of the equation as follows:

(7) $$\begin{array}{c} {\hat{Y}}_{1}\left(t\right)=\left(Y_{0}\left(1\right)+\frac{\beta }{K}\right)e^{K\left(t-1\right)}-\frac{\beta }{K}. \end{array}$$

The final equation is obtained by calculating the score sequence of a student. The minimum solution of the equation is

(8) $$\begin{array}{c} \left(\begin{array}{c} \hat{K}\\ \hat{\beta } \end{array}\right)={\left(B^{T}B\right)}^{-1}B^{T}X, \end{array}$$

in which

(9) $$\begin{array}{c} B=\left[\begin{array}{c} \frac{1}{2}\left[Y_{1}\left(1\right)+Y_{t}\left(2\right)\right.\\ \frac{1}{2}\left[Y_{1}\left(2\right)+Y_{t}\left(3\right)\right.\\ ...\\ \frac{1}{2}\left[Y_{1}\left(N-1\right)+Y_{t}\left(N\right)\right. \end{array}\right]. \end{array}$$

The variable optimal solution of the equation is

(10) $$\begin{array}{c} \lambda =\left(Y_{0}\left(2\right),Y_{0}\left(3\right),...,Y_{0}{\left(N\right)}^{T}\right),\\ Y_{1}\left(i\right)=Y_{1}\left(i-1\right)+Y_{0}{\left(i\right)}^{i}=2,3,...,N. \end{array}$$

Discretize the above formula, bring in the defined variables, and obtain the performance development trend model of physical education learners:

(11) $$\begin{array}{c} {\hat{Y}}_{1}\left(i+1\right)=\left(Y_{0}\left(1\right)+\frac{\hat{B}}{\hat{K}}\right)e^{Ki}-\frac{\hat{B}}{\hat{K}}i=1,2,\ldots . \end{array}$$

According to the formula, it is also necessary to restore the performance prediction process, that is, to obtain the value of the prediction time series model:

(12) $$\begin{array}{c} {\hat{Y}}_{1}\left(i\right)=\left(Y_{0}\left(1\right)+\frac{\hat{B}}{\hat{K}}\right)\left(e^{Ki}-e^{Ki-i}\right)i=1,2,\ldots . \end{array}$$

Finally, test the results of the grey model of physical education learners' performance, and set the relevant error coefficient:

(13) $$\begin{array}{c} \delta \left(i\right)=Y_{0}\left(i\right)-{\hat{Y}}_{0}\left(i\right)i=1,...,N. \end{array}$$

This original grey model is commonly used by most researchers to predict learners' achievement in physical education teaching. On this basis, we combine discrete dynamic modeling technology for optimization. Through the calculation process of the above formula, we find that there are much discrete data in the calculation, which is very helpful to our dynamic modeling. In the discrete dynamic modeling model, we store individual data as subsets in the data system, and each subset will be used many times in processing. Finally, the data effect is analyzed in different cases to obtain the optimal output results. That is to analyze and process the learner's behavior data for many times and select the value with the least repeatability and the least storage for application. In this paper, the accuracy difference between the ordinary grey model and the model optimized by discrete dynamic modeling in the prediction of students' achievement change in physical education teaching is shown in Figure 3.

As can be seen from Figure 3, in the model test, the accuracy of the ordinary grey model decreases significantly with the increase of learner behavior data. Compared with the average prediction accuracy, this paper uses discrete dynamic modeling technology, and the optimized model can maintain the basic accuracy of the model.

## 4. Result Analysis and Discussion

### 4.1. Discrete Dynamic Modeling of Learner Behavior Analysis on Physical Education Teaching Platform

In the analysis of learners' behavior, it mainly involves the following aspects: first, whether each student has prepared before physical education class. The second is the activity of students' online learning and whether they pay attention. Finally, it lies in the situation of watching PE teaching video and students' feedback on video teaching. On the online platform, we control the number of published learning tasks and explore the number of classroom tasks completed by each student. Learners can choose tasks independently according to their own learning needs. Because students' learning environment is different, each student's learning ability is also different, so the data we obtain is discrete and dynamic. The information data faced by traditional modeling technology is static, while discrete dynamic modeling can quickly process dynamic data for effective analysis. In this paper, students of the same grade are randomly selected as experimental variables, and student behavior data are taken as independent variables. The correctness of the efficiency test of traditional modeling technology and discrete dynamic modeling technology for completing tasks is explored, as shown in Figure 4.

In the dynamic data of learners' behavior changes, discrete dynamic modeling technology can accurately grasp the efficiency changes of each student in completing tasks in class. As can be seen from Figure 4, compared with the efficiency of actually completing the task, the efficiency deviation of traditional modeling technology inspection is large. Therefore, in the specific experimental process, students' ability to master physical education teaching knowledge is different.

By setting the theoretical knowledge of topic detection, we can effectively judge students' learning. Before the formal class, according to the learner behavior analysis model, teachers can understand each student's advantages and knowledge points in advance. Therefore, we can judge whether students have a slack learning attitude in the whole classroom.

### 4.2. Analysis of Research Results of Student Achievement Prediction Modeling under the Analysis of Learner Behavior Data in Physical Education Teaching

The data used in the analysis of learners comes from the information produced by the learning process of students in physical education teaching. Data analysis mainly includes collection, acquisition, storage, representation, and other operations. We take the behavior data of college students in physical education classroom as the research content, explore the impact of learners' behavior data on students' performance, and finally predict the trend of students' performance. Through the analysis of students' physical activity records and final scores, teachers can understand the factors affecting students' learning effect in the classroom. Among them, data collection is the most basic part in the prediction process, and it is also the most important link of trend analysis. We use data standards for model construction and use discrete dynamic modeling to process dynamic data. This study obtained the effective class records of more than 9000 learners in the online platform. The data of volleyball, basketball, and tennis in physical education teaching are classified. The specific calculation indicators need to consider the time and overall learning duration of students logging in to the learning platform. Before exploring the factors affecting students' performance, the chaotic and repeated information generated in the data processing process is filtered and screened by discrete dynamic modeling. We ensure that the data obtained is single, simplified, and highly related to physical education teaching. Finally, we need to clean up the data task and delete irrelevant features and recode them. This part of variable data has a great impact on performance prediction.

In the teaching method, we found that the change trend of students' performance through video learning is more obvious. Physical education teachers uploaded 98 video courses in the course, with a total length of 150 minutes. We take students' learning behavior as the monitoring object and select students from two classes to explore. Set the video learning control group. With the increase of learning time, the change of students' performance shows different trends, as shown in Figure 5.

As can be seen from Figure 5, with the increase of learning time, the upward trend of students' performance in general theory teaching is not obvious. The completion rate of students learning through video is about more than 90%, and their grades are obviously rising. Therefore, we preliminarily infer that students' learning situation and enthusiasm are related to learning styles. Most students have high enthusiasm, but in physical education, video learning is more suitable.

## 5. Conclusion

In the big data environment, we use a variety of query methods to analyze the behavior characteristics of learners. Learners' learning ability, emotional attitude, and learning time will affect their performance. In the physical education teaching mode, because its own educational process is different from other disciplines, it needs a large number of practical courses and places as support. The differences of each student's physical quality and learning style will produce corresponding dynamic changes. This paper presents a prediction model based on discrete dynamic modeling technology. This paper analyzes the changing trend of learners' behavior in physical education teaching and its influencing factors on performance. This paper mainly discusses the application of data mining in learner behavior analysis and dynamic data processing. In the learning behavior pattern, feature serialization is used for data encoding. This coding method is a complex data processing process, so we need to carry out effective modeling and analysis after data mining. Secondly, by quantifying the learning process data, the key feature points of students are extracted to provide learners with personalized learning strategies. Compared with the traditional learner behavior analysis model, discrete dynamic modeling can deal with the dynamic information in different environments and improve the overall accuracy of the model. Finally, the dynamic modeling method is used to construct the development and change model of sports performance, and the results of the model are tested. However, the error coefficient and accuracy of the analysis model need to be further discussed. Future research needs to help teachers effectively obtain students' learning state and learning effect on the discrete dynamic modeling of learner behavior analysis.

## Figures and Tables

**Figure 1:** Learner behavior analysis model framework.

**Figure 2:** Dynamic modeling path.

**Figure 3:** Comparison of accuracy between ordinary grey model and optimized model.

**Figure 4:** Comparison between traditional modeling technology and discrete dynamic modeling technology for the correctness of task completion efficiency test.

**Figure 5:** Change trend of students' performance under different modes.

## Data Availability

The data used to support the findings of this study are available from the corresponding author upon request.
